RETRACTED

# Integrated Learning Model-Based Assessment of Enteral Nutrition Support in Neurosurgical Intensive Care Patients

**DOI:** 10.1155/2022/4061043

**Published:** 2022-05-30

**Authors:** Suxue Jiang, Roushi Wang, Haiying Zhang

**Affiliations:** Department of Neurosurgery, East Area 13-a, The First Affiliated Hospital of Suzhou University, Suzhou 215000, China

## Abstract

To observe the clinical efficacy of early enteral nutrition application in critically ill neurosurgical patients, in this paper, we have developed a prediction model for enteral nutrition support in neurosurgical intensive care patients which is primarily based on an integrated learning algorithm. Additionally, we have compared the prediction performance of each model. The patients were divided into control and combined treatment groups according to the random number table method, and 175 patients in each group were treated with a parenteral method and early enteral nutrition support, respectively. A reentry ICU prediction model based on the integrated learning method random forest, adaptive boosting (AdaBoost), and gradient boosting decision tree (GBDT) was developed, and the prediction performance of integrated learning and logistic regression was compared. The average sensitivity, positive predictive value, negative predictive value, false-positive rate, false-negative rate, area under the receiver operating characteristic curve (AUROC), and Brier score after fivefold cross-validation were used to evaluate model effects, and the best performance model based on the top 10 predictor variables in order of importance was given. Among all models, GBDT (AUROC = 0.858) was better than random forest (AUROC = 0.827) and slightly better than AdaBoost (AUROC = 0.851). The GBDT algorithm gave a higher ranking of importance for variables such as mean arterial pressure, systolic blood pressure, diastolic blood pressure, heart rate, urine volume, and blood creatinine and relatively poorer cardiovascular and renal function in neurosurgical intensive care patients.

## 1. Introduction

The nutritional status of neurosurgical intensive care patients is closely related to clinical prognosis. Inadequate nutrition can lead to increased complications, difficulties in ventilator withdrawal, deterioration, prolonged intensive care unit stay, and increased morbidity and mortality [1]. Early gastrointestinal nutrition refers to the supply of daily nutrients required by the patient from the gastrointestinal tract. The main principle is that enteral nutrition should be preferred when the gastrointestinal tract function allows [2]. In our neurosurgery department, 175 patients admitted to the neurosurgical intensive care unit (NICU) were treated with early enteral nutrition support, and good results were obtained and compared with 175 NICU patients treated with traditional parenteral modalities during the same period.

RETRACTED

Neurosurgical critically ill patients are mostly associated with stress hyperglycemia and negative nitrogen balance, and the body is in a hypermetabolic and hypercatabolic state after injury; early enteral nutrition support can improve the nutritional status of patients and enhance their immunity [1] but is prone to complications such as feeding intolerance and aspiration pneumonia [2]. To achieve better care outcomes, evidence-based care is derived from evidence-based medical theory by integrating the best available evidence-based medical evidence, the patient's actual situation, and the caregiver's skills and clinical experience [3, 4].

In this paper, we have developed a prediction model for enteral nutrition support in neurosurgical intensive care patients, which is based on an integrated learning algorithm, and compared the prediction performance of each model. The patients were divided into control and combined treatment groups according to the random number table method, and 175 patients in each group were treated with parenteral approach and early enteral nutrition support, respectively. Prediction models for readmission to ICU were developed based on integrated learning method random forest, adaptive boosting (AdaBoost), and gradient boosting decision tree (GBDT), and the prediction performance of integrated learning and logistic regression was compared. Among all models, GBDT (AUROC = 0.858) outperformed random forest (AUROC = 0.827) and was slightly better than AdaBoost (AUROC = 0.851). Compared with logistic regression (AUROC = 0.810), the integrated learning algorithm has a greater improvement in the discrimination.

## 2. Objects and Methods

### 2.1. Research Subject

The 350 patients admitted to the NICU were divided into control and combined treatment groups according to the random number table method, and 175 patients in each group were treated with a parenteral method and early enteral nutrition support. All patients are screened for nutritional risk. No one was excluded through exclusion criteria.

Both groups were given routine nursing interventions for neurosurgical intensive care patients, including psychological interventions, medication guidance, infection prevention, and rehabilitation training. In the control group, patients were also given conventional nutritional support, including parenteral nutrition support (24 h after injury) and enteral nutrition support (48 h after injury or after the recovery of postoperative bowel sounds), while the experimental group was given enteral nutrition support based on the evidence-based concept.

RETRACTED

Establish an evidence-based nursing intervention team including a nurse manager, an attending physician, and 7 nurses; organize learning about neurosurgical critical illness, nutrition support, evidence-based nursing, etc.; and identify evidence-based issues around the focus of this study such as duration of enteral nutrition support, nutrition route, nutrition methods, and complication prevention.

Inclusion criteria are as follows:

1. All were diagnosed by brain CT or MRI as cerebral contusion, intracranial hematoma, or brainstem injury
2. Glasgow coma score of ≤8 points
3. The onset to treatment time ≤ 12 h and Nutrition Risk Screening (NRS 2002) ≥ 3

Exclusion criteria are as follows:

1. With dysfunction of important organs
2. With endocrine diseases

#### 2.1.1. Duration of Enteral Nutrition Support

- *Evidence-Based Support*. Neurosurgical critically ill patients are mostly associated with stress and impaired consciousness, which can lead to dysphagia and a high catabolic state of the organism. Early enteral nutrition support can help maintain the intestinal barrier function, improve the metabolic state of the body, and enhance immunity [5]
- *Early Nutritional Support*. Enteral nutrition solution (Beprid) is given 24 h after injury or surgery, along with a progastric motility drug (Gastroflucan)

#### 2.1.2. Nutritional Approach

- *Evidence-Based Support*. To enhance nutritional risk assessment and control the rate of nutrient drip according to patients' energy metabolism differences [6]
- *Nursing Interventions*. Calculate basal energy expenditure and daily energy expenditure [7]. On day 1, 20 ml/h, supplying 500 kcal/d; on days 3-5, 30-50 ml/h, supplying 25-30 kcal/(kg-d), with energy deficiency supplemented by parenteral nutrition; after day 5, 80-100 ml/h, supplying 25-30 kcal/(kg-d), with complete enteral nutrition. On day 1, protein 1.2 g/(kg·d) calculated the standard dose for each patient, starting at 10 ml/h continuous instillations, increasing the dose by 10 ml every 12 h as shown in Table 1

#### 2.1.3. Nutrition Route

- *Evidence-Based Support*. Enteral nutrition is prone to complications such as reflux, misaspiration, and aspiration pneumonia [8], and the incidence of gastric retention, misaspiration, and pneumonia is significantly higher in the nasogastric tube enteral nutrition than in the nasogastric tube group [9–11]
- *Nursing Intervention*. Using the nasogastric tube placement method, the patient was placed in a semirecumbent position, the nasogastric tube insertion length was measured, the guiding wire was inserted into the nasogastric tube, and the nasogastric tube was slowly inserted from the nasal cavity to the target position (110-120 cm in men and 105-110 cm in women), and the adhesive tape was fixed to the tip of the nose. Chest radiograph was used to determine the position of the intestinal tube

The complication prevention is as follows:

1. *Evidence-Based Support*. Early nutritional support in neurosurgical intensive care patients is prone to various complications such as nausea, vomiting, and aspiration errors, which are the main causes of feeding intolerance [12]
2. *Nursing Interventions*. Assess the patient's degree of impaired consciousness and choking reflex before feeding and develop an individualized diet according to the situation; determine the position of the gastric or intestinal tube before nasal feeding
3. Elevate the head of the bed ≥ 30° if there is no contraindication during feeding; maintain a stable nasal drip rate and adhere to the principle of starting with a small dose (20 ml/h); use gastric motility drugs appropriately; give the patient abdominal massage after feeding
4. Transfer the patient or will perform a lumbar puncture, extubation of tracheal intubation, and other
5. Gently perform operations such as suctioning and turning
6. Suspend nasal feeding with the head tilted to one side when vomiting
7. Give gastrodynamic drugs when abdominal distension and poor digestion occur
8. Perform swallowing and respiratory exercises as early as possible
9. Give patients who have not relieved their stools for more than 3 days and give 40 ml of RECT to patients who have not relieved stool for more than 3 days
10. Enteral nutrient solution (perplex) is given after injury or 24 hours after surgery, along with gastric motility agents (gastric reassurance) as shown in Table 2

Prior to modeling, feature selection was performed in this study to find the best combination of predictor variables using recursive feature elimination based on logistic regression. The recursive feature elimination results showed that the predictive performance of the model increased while the number of features was increasing (Figure 1). Therefore, the recursive feature elimination method based on logistic regression suggests that all the features incorporated in this study contribute to the prediction effect of the model. If only some of the features are selected, it may lead to a decrease in the prediction performance of the model, so all the features are incorporated in this study, and no selection of features is made to ensure the best prediction performance.

RETRACTED

## 3. The Proposed Prediction Model

In logistic regression, the dependent variable is dichotomous, and the posterior probability of a sample falling into a category is modelled as a logit function without prior assumptions about the data distribution (Figure 2). The logit function can be used to transform the linear combination of independent variables into predicted values between 0 and 1, to obtain the probability of occurrence of a certain category of events, and to determine the category of the outcome based on the probability magnitude, which is widely used because of its high interpretability.

Random forest mainly uses a parallel method of bagging for integrated learning, using a decision tree as the base classifier, with the independent variable *x* corresponding to the node feature variables in the decision tree model and the dependent variable *y* corresponding to the leaf node variable values in the decision tree (Figure 3). In the training process of the random forest, firstly, by bootstrap method, there are randomly put-back sampling *N* times from *N* training sample data sets, and some of the samples will be duplicated, and the proportion of samples that are always not sampled in *N* times is 1 − 1 − 1( )*NN*, and when *N* is taken as the limit, about 36.8% of the overall samples will not appear in the sampling set. The proportion of samples that do not appear in the sample set is 1 − 1 − 1() *NN*, and when *N* is taken as the limit, about 36.8% of the overall sample will not appear in the sample set. In addition, the randomness of the random forest is also reflected in the random feature selection. In the process of training the base classifier with the sampled sets, a subset of *k* features is randomly selected from the overall features, the features with the smallest Gini impurity are selected from the subset, and the current decision tree node is determined. One base classifier is trained for each sampled set to form the final random forest model, and when using this model to make classification decisions, *T* base classifiers vote to determine the classification result.

AdaBoost is a representative algorithm of integrated learning boosting (boosting), which uses the base classifier single-layer decision tree for serial training to obtain a stronger classifier. In each training round, the error rate *e*_*m*_ of the current base classifier (*m* is the number of iterations, *m* = 1, 2, ⋯, *M*) is used to determine the base classifier weights *a*_*m*_ for the current round, while the sample weights are updated and the next base classifier is trained based on the new sample weights *G*_*m*+1_(*x*), and the final output of AdaBoost is a weighted combination of all base classifiers.

First, calculate the classification error rate of the base classifier on the training set:

(1) $$\begin{array}{c} e_{m}=P\left(G_{m}\left(x_{i}\right)\neq y_{i}\right)=\overset{N}{\underset{i=1}{\sum }}w_{mi}I\left(G_{m}\left(x_{i}\right)\neq y_{i}\right),i=1,2,\cdots ,N, \end{array}$$

where *N* is the total number of samples, *w*_*mi*_ is the weight of the *i*th sample in the *m*th iteration, and *I* represents the indicator function that results in 0 or 1. When training the first base classifier *G*_*I*_, equal weights are assigned to the *N* training samples. The larger the error rate of a classifier, the smaller its weight in the final model, and the weight of each classifier is determined based on the error rate of the classifier *a*_*m*_.

(2) $$\begin{array}{c} \alpha_{m}=\frac{1}{2}\ln\left(\frac{1-e_{m}}{e_{m}}\right). \end{array}$$

At the same time, the weights of the training samples are updated, and higher weights are assigned to the misclassified samples:

(3) $$\begin{array}{c} w_{m+1,i}=\frac{w_{m,i}}{Z_{m}}\exp\left(-\alpha_{m}y_{i}G_{m}\left(x_{i}\right)\right)\;i=1,2,\cdots ,N, \end{array}$$

where *Z*_*m*_ is the normalization factor, calculated as follows:

(4) $$\begin{array}{c} Z_{m}=\overset{N}{\underset{i=1}{\sum }}w_{m,i}\exp\left(-\alpha_{m}y_{i}G_{m}\left(x_{i}\right)\right). \end{array}$$

Next, the next basic classifier *G*_*m*+1_(*x*)(*m* + 1 ≤ *M*) is trained, and a new basic classifier is generated in each iteration to best fit the current weighted sample. The output of AdaBoost is the weighted combination of the results of each basic classifier, and the formula is as follows:

(5) $$\begin{array}{c} f\left(x\right)=\overset{M}{\underset{m=1}{\sum }}\alpha_{m}G_{m}\left(x\right). \end{array}$$

The final classification result is obtained by judging the probability of *F* (*x*) output.

RETRACTED

GBDT is an improved boosting algorithm. Taking classification and regression tree (CART) as the basic classifier, a series of carts are connected in series to obtain an integrated learning model.

At the beginning of training, all samples *X* have the same initialization *F*_0_(*x*). In *M* (*M* = 2, 3, ⋯, *m*), in the process of the next iteration, calculate the residual *F*_*m*−1_(*x*) between the predicted value ${\hat{y}}_{i}$ and the real value of the model, then establish the residual of the cart fitting model, and finally combine the output of ${\hat{y}}_{i}$ and cart to obtain a new round of prediction model *F*_*m*−1_(*x*), where the residual ${\hat{y}}_{i}$ between the predicted value and the real value of the model is approximated by the negative gradient of the loss function relative to *F*_*m*−1_(*x*). With each iteration of GBDT, the fitting error will be reduced. The main prediction outcome of this study is the binary variable, and the loss function of GBDT for the binary problem is defined as follows:

(6) $$\begin{array}{c} L\left(y,F\left(x\right)\right)=\ln\left(1+\exp\left(-2yF\left(x\right)\right)\right),y\in \left\{-1,1\right\}, \end{array}$$

where *f* (*x*) is as follows:

(7) $$\begin{array}{c} F\left(x\right)=\frac{1}{2}\ln\left[\frac{\mathrm{Pr}\left(y=1\left|x\right.\right)}{\mathrm{Pr}\left(y=-1\left|x\right.\right)}\right]. \end{array}$$

The ultimate goal of GBDT model is to find *f*(*x*) that minimizes the loss function (7) and then calculate the prediction probability of samples to obtain the results of sample classification. Establish a two-class GBDT model. Firstly, initialize the GBDT model according to the following:

(8) $$\begin{array}{c} F_{0}\left(x\right)=\frac{1}{2}\ln\left(\frac{N_{y+}}{N_{y-}}\right). \end{array}$$

In the next GBDT model iteration, in order to minimize the loss function of each iteration, it is necessary to move towards the negative gradient of the loss function during each iteration. The negative gradient ${\hat{y}}_{i}$ of the *M* (*M* = 2, ⋯, *m*) iteration is the approximation of the residual between the predicted value *F*_*m*−1_(*x*) and the real value *y*_*i*_ of the model in the previous iteration:

(9) $$\begin{array}{c} {\tilde{y}}_{i}=-{\left[\frac{\partial L\left(y_{i},F\left(x_{i}\right)\right)}{\partial F\left(x_{i}\right)}\right]}_{F\left(x\right)=F_{m-1}\left(x\right)}=\frac{2y_{i}}{\left(1+\exp\left(2y_{i}F_{m-1}\left(x_{i}\right)\right)\right)},i=1,2\cdots_{N}. \end{array}$$

Then, a new training data set ${\left\{x_{i},{\tilde{y}}_{i}\right\}}_{1}^{N}$ is formed by using the sample data *x*_*i*_ and the negative gradient value ${\hat{y}}_{i}$ calculated by formula (9), *N*1 (*n* is the number of samples), a cart model {*R*_*jm*_}_1_^*J*^ with *J* termination nodes (leaf nodes) is trained, and the value of cart leaf nodes is further calculated:

(10) $$\begin{array}{c} \gamma_{jm}=\frac{\sum_{x_{i}\in R_{jm}}{\tilde{y}}_{i}}{\sum_{x_{i}\in R_{jm}}\left|{\tilde{y}}_{i}\right|\left(2-\left|{\tilde{y}}_{i}\right|\right)},j=1,2\cdots J. \end{array}$$

After obtaining the output of the new basic classifier, the current model *F*_*m*_(*x*) of GBDT can be obtained by concatenating the output result of cart with the previous round model *F*_*m*−1_(*x*):

(11) $$\begin{array}{c} F_{m}\left(x\right)=F_{m-1}\left(x\right)+\overset{J}{\underset{j=1}{\sum }}\gamma_{jm}I\left(x\in R_{jm}\right). \end{array}$$

The predicted probability value of the final model is as follows:

(12) $$\begin{array}{c} \mathrm{Pr}\left(y=1\left|x\right.\right)=\frac{1}{1+\exp\left(-2F_{m}\left(x\right)\right)}. \end{array}$$

RETRACTED

## 4. Results and Observations

### 4.1. Comparison of Serum Nutritional Indexes between the Two Groups before and after Intervention

Before the intervention, there was no significant difference in the contents of serum ALB and Hb between the two groups (*P* > 0.05). The overall analysis showed that there were significant differences in the contents of serum ALB and Hb between the two groups, time point, and interaction (all *P* < 0.05). Further comparison between the two groups showed that the contents of serum ALB and Hb in the two groups were significantly lower than those in the same group before intervention for 1 and 2 weeks, the contents of serum ALB and Hb in the two groups were significantly higher than those in the same group for 1 week (*P* < 0.05), and the contents of serum ALB and Hb in the experimental group were significantly higher than those in the control group for 1 and 2 weeks (*P* < 0.05), see Table 3.

### 4.2. Comparison of Complications between the Two Groups

The incidence of gastrointestinal dysfunction in the experimental group was significantly lower than that in the control group (*P* < 0.05). There were 8 cases of pulmonary infection and 6 cases of urinary infection in the experimental group and 11 cases of pulmonary infection and 9 cases of urinary infection in the control group. There was no significant difference in the infection rate between the two groups (*P* > 0.05), see Table 4.

### 4.3. Comparison of Prognosis between the Two Groups

The prognosis of the experimental group was significantly better than that of the control group (*P* < 0.05), see Table 5.

### 4.4. Model Performance

An ensemble learning algorithm is one of the best algorithms for fitting structured data at present. This study mainly establishes the risk prediction model of patients' reentry into ICU based on an ensemble learning algorithm and compares the prediction effects of various models. Compared with logistic regression, which is widely used in the biomedical field, the ensemble learning model has better prediction performance. Compared with the reported risk prediction model of reentry into ICU, the prediction model in this study has higher discrimination and can better predict the risk of reentry into ICU. Early identification of high-risk patients is helpful for clinicians to make better medical decisions as shown in Figure 4.

In this study, two data balancing algorithms are used for data preprocessing. Compared with random downsampling, near-miss method improves the performance of the model better. In the process of processing samples, random downsampling loses a large number of information of most kinds of samples, which has the problem of insufficient representation of samples. Through the *k*-nearest neighbor algorithm, the near-miss method selects the most class samples closest to the few class samples, which better retains the decision boundary of the original samples. Therefore, it is more representative than the samples sampled at random, and the improvement of the model is more significant.

RETRACTED

## 5. Discussion

Early enteral nutrition support applied to severe neurosurgical patients can improve patients' metabolic status, regulate immune function, maintain the integrity of gastrointestinal mucosal function and structure, prevent secondary injury, and then reduce the disability rate and mortality of severe patients. The key problem is how to safely and effectively give early enteral nutrition support.

There is much literature about early enteral nutrition in severe neurosurgical patients, but the starting time, nutritional path, and nutritional method of enteral nutrition support are still controversial. Relevant guidelines and literature point out that, if intestinal function permits, enteral nutrition after injury or 24~48 hours after the operation is helpful to maintain intestinal barrier function. According to the difference of patients' energy metabolism, giving patients the necessary energy supply can ensure patients' nutritional status and improve immunity. It is difficult to implement these measures. Evidence-based nursing puts forward specific and structured evidence-based problems through the analysis of the impact of various factors, collects 1 ~ 4 types of the empirical literature, obtains evidence-based support through careful evaluation, and formulates evidence-based nursing intervention plan in combination with the clinical experience and skills of nurses, which can ensure the pertinence and accuracy of nursing intervention.

This study carried out evidence-based research on the four key nodes of enteral nutrition support time, nutrition pathway, nutrition method, and complication prevention. Enteral nutrition support was given after self-injury or 24 hours after the operation. The international general energy calculation method was used to ensure the energy supply at different time points; the nasointestinal tube was used as the nutrition support pathway, supplemented by comprehensive complication prevention measures. The results showed that serum ALB and Hb in the experimental group were significantly higher than those in the control group at 1 and 2 weeks of intervention, suggesting that early enteral nutrition support based on the evidence-based concept can improve the nutritional status of severe neurosurgical patients. The start time of 48 h enteral nutrition support in patients with severe craniocerebral injury was positively correlated with the improvement of neurological function and survival rate. The function of the small intestine of critically ill patients in the department of neurosurgery is relatively normal. The nasointestinal tube through the stomach pylorus directly to the duodenum and jejunum can effectively prevent complications such as reflux, gastric retention, and aspiration pneumonia and improve the enteral nutrition support tolerance [9]. Head elevation of 20° ~30° is an effective method to prevent reflux. Controlling the temperature of the feeding solution and maintaining stable infusion speed are important measures to protect gastrointestinal function and prevent infection. Nursing intervention guided by evidence-based concept analyzes and integrates these nursing measures supported by evidence-based medicine and applies them to early enteral nutrition support for severe patients in neurosurgery, which can ensure the safety of enteral nutrition support. The results showed that the incidence of gastrointestinal dysfunction in the experimental group was significantly lower than that in the control group, and the prognosis was significantly better than that in the control group. Zhan Yuxin et al. also reported similar results.

RETRACTED

In conclusion, the application of nursing intervention based on an evidence-based concept in enteral nutrition support for severe neurosurgical patients can improve the nutritional status of patients, reduce the incidence of complications, and improve the prognosis of patients.

## 6. Conclusion and Future Work

In this paper, a prediction model of enteral nutrition support for severe neurosurgical patients is established based on an integrated learning algorithm, and the prediction performance of each model is compared. The NICU patients in our hospital were selected as the research object. The prediction model was established based on the integrated learning method random forest, adaptive lifting algorithm, and gradient lifting decision tree, and the prediction performance of integrated learning and logistic regression was compared. Ensemble learning algorithm has a great improvement in discrimination. In the order of importance of variables given by GBDT algorithm, mean arterial pressure, systolic blood pressure, diastolic blood pressure, heart rate, urine output, blood creatinine, and other variables rank first. Relatively speaking, cardiovascular function and renal function of neurosurgical critically ill patients are worse.

The proposed model can be made more effective if state-of-the-art existing approaches were integrated with it. Moreover, the prediction accuracy can be further improved if the training process of the model is based on artificial intelligence.

RETRACTED

## Figures and Tables

**Figure 1:** Recursive feature elimination method based on logistic regression.

**Figure 2:** Schematic diagram of the logit function.

**Figure 3:** Schematic diagram of the decision tree.

**Figure 4:** Comparison of different ensemble learning methods.

**Table 1:** Comparison of general information between the two groups.

Group	Number of cases	Gender (example, male/female)	Age (years)	Damage type (case)				Treatment methods (cases)	GCS $\bar{x}\pm s$
				Brain contusion	Intracranial hematoma	Brain stem injury	Operation	Conservative	
Experience group	72	42/30	48.52 ± 6.24	31	26	15	70	2	6.35 ± 1.12
Control group	64	43/21	47.38 ± 6.18	30	20	12	6	2	6.48 ± 1.20
*x* ^2^/*t* value		1.133	1.068		0.388		0.014		0.653
*P* value		0.287	0.287		0.824		0.905		0.515

**Table 2:** Performance of random downsampling and near-miss methods for unbalanced data.

Classifier	Random undersampling	Accuracy
		Near-miss
Logistic regression	0.615	0.838
Random forest	0.542	0.844
AdaBoost	0.620	0.873
GBDT	0.626	0.874

**Table 3:** Comparison of serum nutritional indexes between the two groups before and after intervention (g/l) $\bar{x}\pm s$.

Group	Number of cases	ALB	Hb
Experience group	72		
Before intervention		36.84 ± 4.32	123.52 ± 14.33
Intervention 1 week		32.54 ± 4.39	110.07 ± 10.34
Intervention 2 weeks		35.34 ± 3.04	118.58 ± 7.18
Control group	64		
Before intervention		30.31 ± 3.28	101.36 ± 7.95
Intervention 1 week		32.64 ± 4.02	110.49 ± 6.48
Intervention 2 weeks		36.99 ± 5.40	127.00 ± 13.64

**Table 4:** Comparison of complications between the two group (cases (%)).

Group	Number of cases	Gastrointestinal dysfunction	Infected
Experience group	72	8 (11.11)	14 (19.44)
Control group	64	17 (26.56)	20 (31.25)
*x* ^2^ value		5.392	2.519
*P* value		0.020	0.113

**Table 5:** Comparison of prognosis between the two groups (cases (%)).

Group	Number of cases	The prognosis is good	Medium disability	Severe disability or plant survival	Death
Experience group	72	24 (33.33)	26 (33.33)	22 (30.56)	0
Control group	64	11 (17.18)	26 (28.13)	nnn (42.19)	0
*Z* value	4.885				
*P* value	0.087				

## Data Availability

The datasets used and analyzed during the current study are available from the corresponding author upon reasonable request.
